RETRACTED

# Quercetin-induced miR-200b-3p regulates the mode of self-renewing divisions in pancreatic cancer

**DOI:** 10.1186/s12943-017-0589-8

**Published:** 2017-01-31

**Authors:** Clifford C. Nwaeburu, Alia Abukiwan, Zhefu Zhao, Ingrid Herr

**Affiliations:** Department of General, Molecular OncoSurgery, Section Surgical Research, Visceral and Transplantation Surgery, University of Heidelberg, Im Neuenheimer Feld 365, 69120 Heidelberg, Germany

## Abstract

**Background:**

Cancer stem cells are suggested to contribute to the extremely poor prognosis of pancreatic ductal adenocarcinoma and dysregulation of symmetric and asymmetric stem cell division may be involved. Anticancer benefits of phytochemicals like the polyphenol quercetin, present in many fruits, nuts and vegetables, could be expedited by microRNAs, which orchestrate cell-fate decisions and tissue homeostasis. The mechanisms regulating the division mode of cancer stem cells in relation to phytochemical-induced microRNAs are poorly understood.

**Methods:**

Patient-derived pancreas tissue and 3 established pancreatic cancer cell lines were examined by immunofluorescence and time-lapse microscopy, microRNA microarray analysis, bioinformatics and computational analysis, qRT-PCR, Western blot analysis, self-renewal and differentiation assays.

**Results:**

We show that symmetric and asymmetric division occurred in patient tissues and in vitro, whereas symmetric divisions were more extensive. By microarray analysis, bioinformatics prediction and qRT-PCR, we identified and validated quercetin-induced microRNAs involved in Notch signaling/cell-fate determination. Further computational analysis distinguished miR-200b-3p as strong candidate for cell-fate determinant. Mechanistically, miR-200b-3p switched symmetric to asymmetric cell division by reversing the Notch/Numb ratio, inhibition of the self-renewal and activation of the potential to differentiate to adipocytes, osteocytes and chondrocytes. Low miR-200b-3p levels fostered Notch signaling and promoted daughter cells to become symmetric while high miR-200b-3p levels lessened Notch signaling and promoted daughter cells to become asymmetric.

**Conclusions:**

Our findings provide a better understanding of the cross talk between phytochemicals, microRNAs and Notch signaling in the regulation of self-renewing cancer stem cell divisions.

**Electronic supplementary material:**

The online version of this article (doi:10.1186/s12943-017-0589-8) contains supplementary material, which is available to authorized users.

## Background

Pancreatic Ductal Adenocarcinoma (PDA) is a highly malignant tumor with late diagnosis and poor prognosis [1]. The tumors are believed to proliferate rapidly, re-occur, be resistant or result in metastasis with cancer stem cells (CSCs) as main responsive mediator [2]. CSCs may be potential diagnostic and therapeutic targets because of their roles in carcinogenesis [3]. CSCs are known for their self-renewing and/or differentiation potential [4]. CSC self-renewing division gives rise to symmetric or asymmetric cell division. The former, resulting to two identical daughter cells and the later to two dissimilar daughter cells [5]. Asymmetric division is performed by CSCs for homeostasis [6] while symmetric division results in exponential tumor growth [7].

RETRACTED

Studies have shown different regulators of the CSCs mode of divisions [8]. Notable amongst them is the Notch signaling pathway [9–11]. It is a highly dysregulated pathway in cancer [12]. Notch is an essential gene encoding a signaling receptor, which has a major contribution to proper development, cell fate decision, cell proliferation and survival [13, 14]. Notch is suggested as marker for symmetric cell division and oncogene [10, 15, 16]. Notch inhibitor [17], Numb, is a cell fate determinant [18] and implicated as a tumor suppressor [19] and marker for asymmetric cell division [20].

Via the modulation of the Notch signaling pathway, microRNAs (miRs) have been identified to play a major role in CSCs fate determination [21, 22]. MiRs are small non-coding RNAs that functions in RNA silencing and post transcriptional regulation of gene expression [23]. MiR therapy therefore offers an attractive anti-tumor approach. Recently, we have shown that the anti-cancer phytochemical, quercetin, regulates the expression of miRs in PDA via Notch signaling [24].

Quercetin is a flavonoid obtained from plant sources such as leafy vegetables, onions, apples, black tea and nuts [25]. However, irrespective of the importance of quercetin modulation of miR signaling in PDA and miR-mediated role in CSCs fate determination via the Notch signaling pathway, it remains unknown whether an individual quercetin-induced miR plays any role in the regulation of the mode of self-renewing divisions in PDA.

Here, we show that, both symmetric and asymmetric modes of division occur in PDA with symmetric division mostly occurring, especially at the principal sites of three proliferation and asymmetric division at the periphery. This phenomena results to exponential proliferation, increase in the levels of Notch and decrease in Numb levels. Using miR profiling, we show that miR-200b-3p is upregulated after quercetin treatment of PDA cells. In silico analyses suggests miR-200b-3p as a cell fate determinant miR in PDA as it is predicted to target the segregating determinants in human. MiR-200b-3p is shown to switch the mode of CSCs division from symmetric to asymmetric division by inhibiting Notch and activating Numb. This observation is further reinforced by time-lapse microscopy analysis. Investigation of CSCs self-renewal in vitro, demonstrated a vital role for miR-200b-3p to inhibit CSCs self-renewal and subsequently, induce osteogenic, adipogenic and chondrogenic differentiations. These studies offer new insights into the mode of self-renewing CSCs divisions, underscoring the distinctive regulatory functions accomplished by miRs.

RETRACTED

## Methods

### Tumor cell lines

Pancreatic cancer established cell lines; AsPC1 and PANC1 were obtained from the American Type Culture Collection (Manassas, VA, USA) and recently authenticated by a commercial service (Multiplexion, Heidelberg, Germany). The human, primary pancreatic cancer cell line ASANPaCa was generously provided by Dr. Nathalia Giese and is described [26]. Frozen stocks were prepared from initial stocks, and every 3 months a new frozen stock was used for experiments in order to maintain the authenticity of the cell lines. Monthly examination ensured mycoplasma negative cultures. Cells were cultured in DMEM (PAA, Pasching, Austria) supplemented with 10% heat-inactivated FCS (Sigma, Deisenhoffen, Germany) and 25 mmol/L HEPES (PAA, Pasching, Austria).

### Cell synchronization

All cells were synchronized prior to any experiment by serum starvation as previously described [27, 28]. The cells were seeded with 10% FCS culture medium on the first day. On the second day, the medium was removed and the cells synchronized with 0.1% FCS culture medium for 24 h.

### Tumorsphere forming assay and analysis

PDA cells were resuspended in tumorsphere DMEM/F12 medium (Thermo Fisher Scientific Inc., Dreieich, Germany) supplemented with B27 supplement (50×) (Thermo Fisher), 20 ng/mL rEGF (Thermo Fisher), 20 ng/mL bFGF (Thermo Fisher), 5 μg/mL I nsulin (Sigma, Deisenhoffen, Germany) and 5 mL Glutamax (Thermo Fisher). To avoid false positives as a result of cell aggregation, 1000 cells in 50 μL tumorsphere medium mixed with 50 μL matrigel were cultured per well of a 24-well plate. The mixture was allowed to polymerize for 1 h at 37 °C and 5% CO_2_. Subsequently, 1 mL of the tumorsphere medium was added per well, either alone or supplemented with 50 nM *mir*Vana™ mimics or 50 μM quercetin. Seventy-two hours later, the spheres were collected by gentle centrifugation, dissociated into single cells, and cultured for the formation of next generation spheres. Tumor spheres were counted using an inverted microscope (Nikon Eclipse TS100; Nikon GmbH, Düsseldorf, Germany). To quantify cell numbers, the tumor spheres were collected and disassociated with Trypsin-EDTA (Thermo Fisher) to make a single cell suspension. The viable cells were then counted using the Z™ Series COULTER COUNTER® Cell and Particle Counter (Beckman Coulter, Indianapolis, USA).

RETRACTED

### Time-lapse microscopy

Cells were plated at low density in μ-Dish 35 mm (Ibidi, Germany) and placed in the Nikon BioStation IM-Q (Nikon Instruments Europe) compact cell incubator and monitoring system. Cells were photographed every 30 min for about 80 h. The microscope was equipped with an incubator that maintains the temperature at 37 °C, a humidifier that maintains a humidity level of 95% and a stable CO_2_ flow of 5%. Time-lapse sequences were combined using FIJI software.

### Evaluation of differentiation to adipocytes

Cells were seeded at a density of 4.5 × 10^4^ cells/well in 6-well cell culture plates. At about 90% cell density, cells were left untransfected, treated with 50 μM quercetin or were transfected with 50 nM *mir*Vana™ mimics of miR-200b-3p or a miR-NC (Thermo Fischer Scientific, Waltham, MA USA) using lipofectamine RNAiMax reagent (Life Technologies, Darmstadt, Germany) for every 72 h for a period of 12 days. The cells were washed with PBS, fixed with methanol for 5 min at room temperature and incubated with Oil Red O staining reagent for 20–30 min on a plate shaker at room temperature. Afterwards, the cells were washed with deionized water. Heterogeneous adipocytes are stained red by the Oil Red O staining solution and visualized with a 10× magnification using an inverted microscope (Nikon Eclipse TS100; Nikon GmbH, Düsseldorf, Germany).

### Evaluation of differentiation to osteoblasts

Cells were seeded and treated as described above. The cells were washed with PBS, fixed with 10% neutral buffered formalin for 60 s and incubated in the dark with FAST BCIP/NBT (Sigma) for 10–20 min. Afterwards, cells were washed with deionized water. Heterogeneous alkaline phosphatase expressed by osteoblasts develops the NBT substrate into deep bluish purple color.

### Evaluation of differentiation to chondrocytes

Cells were seeded and treated as described above. The cells were washed with PBS and fixed with 10% neutral buffered formalin for 60 min at room temperature. After two rounds of washing with distilled water, the cells were incubated overnight in the dark at room temperature with Alcian blue staining solution (Sigma-Aldrich, St. Louis, Missouri, USA). Heterogeneous chondrogenic differentiation was identified as intense dark-blue coloration due to the formation of aggrecan.

### Western blot analyses

Western blot analyses were done as formerly described [29]. Antibodies used include: rabbit antibodies against human Notch (Cell Signaling Technology, Danvers, USA), Numb (Cell Signaling Technology, Danvers, USA) (Cell Signaling Technology, Danvers, USA), and β-actin (Sigma-Aldrich, St. Louis, Missouri, USA).

RETRACTED

### Patient tissue

Patient materials were obtained under the approval of the ethical committee of the University of Heidelberg after receiving written informed consent from the patients. The diagnoses were established by conventional clinical and histological criteria according to the World Health Organization (WHO). All surgical resections were indicated by the principles and practice of oncological therapy.

### Immunohistochemical and Immunofluorescence staining

Staining was done on 6-μm frozen tissue sections or in established cell lines as previously described [29, 30].

### MicroRNA transfection

MirVana™ mimics (miR-200b-3p and miR-NC) (Thermo Fisher Scientific Inc., Dreieich, Germany), 50 nM each, were transfected into the cells using Lipofectamine 2000 (Thermo Fisher) or Lipofectamine RNAiMAX transfection reagent (Thermo Fisher) with the reverse transfection method as described in the manufacturer’s instructions.

### Dual-Luciferase® reporter assay

Cells were seeded at a density of 1 × 10^4^ cells per well of a 96-well plate and co-transfected with 50 nM miR mimics, 25 ng/well of firefly luciferase plasmid and 50 ng/well renilla luciferase reporter construct expressing Notch1 3‘UTR (BioCat, Heidelberg, Germany). The cells were lysed in Passive Lysis Buffer of the Dual Luciferase® Assay System (Promega, Mannheim, Germany) at 48 h post-transfection. Renilla and firefly luciferase (Promega) activities were measured on the FLUOstar OPTIMA instrument (BMG Labtech, Ortenberg, Germany).

### MicroRNA Microarray profiling and analyses

This was performed using the Agilent Human miRNA Microarray (Release 19.0) as previously described [24].

### MicroRNA *in silico* analyses

The miRNA gene targets’ predictions based on miRanda and TargetScan and PicTar were downloaded from http://www.microrna.org [31], http://www.targetscan.org [32] respectively. “Good” mirSVR score refers to miRNA targets with < −0.1 score, and “non-good” mirSVR score refers to targets with > −0.1 score obtained from the support vector regression algorithm mirSVR, available with miRanda predictions from http://www.microrna.org.

### Taqman miRNA RT-qPCR

This was done as previously described [24]. cDNA was prepared from 500 ng total RNA using the Taqman® Reverse Transcription Reagents (Thermo Fisher Scientific, Dreieich, Germany) in accordance to the manufacturers’ instructions. Quantitative levels of hsa-miR-200b-3p were measured from 1 μl of synthesized cDNA using their respective primer assays and RNU44 as endogenous control (Applied Biosystems, Darmstadt, Germany). Notch1 and Numbl mRNA levels were quantified from 2 μl of synthesized cDNA using the TaqMan Gene Expression Assay and primers for Notch1, Numbl and GAPDH (Thermo Fisher Scientific). StepOne Real-Time PCR System (Applied Biosystems) was used for the PCR. Changes in the relative concentration were calculated with the second derivative maximum method 2^−ΔCT^. ΔCT was calculated by subtracting the CT of the housekeeping gene from the CT of the gene of interest. The fold change was obtained by the equation 2^−ΔΔCT^.

RETRACTED

### Statistical analyses

The quantitative data are presented as the mean ± SD. The data were analyzed using Student’s *t*-test for statistical significance. *P* < 0.05 was deemed to be statistically significant.

## Results

### Symmetric Cell Division (SCD) mostly occurs in PDA cells

It is an established fact that CSCs divide by both symmetric and asymmetric cell divisions [5] with asymmetric division maintaining suitable numbers of cell offspring [6] and symmetric division, imperative for growth and regenerative competences [7]. In addition, Notch and Numb genes are crucial to self-renewing divisions as markers for symmetric and asymmetric division markers respectively [5] (Fig. 1a). Hence, we set out to identify the mode of CSCs divisions occurring in PDA. To this end, firstly, we performed immunofluorescence analysis using PDA patient samples, staining for Notch and Numb. The expression of Notch was observed to be more than Numb. Notch expressions were found mostly at the pancreatic ductal glands, while Numb was mostly expressed at the periphery (Fig. 1b). This observation was verified by double immunofluorescence staining of the ductal marker, cytokeratin with notch; cytokeratin with numb and the human proliferation marker, Ki67 with Notch (Additional file 1: Figure S1). Secondly, we performed time-lapse microscopy, monitoring synchronized single PDA cells from the established and CSC-enriched cell lines AsPC1 and PANC1 [33] for a period of 3 consecutive divisions. Studies show that a cell divides symmetrically, if its first three divisions results to 2, 4 and 8 cells respectively, and asymmetrically if it is 2, 3 and 5 cells instead [7, 34] (Fig. 1c). Our results show that the cells were mostly undergoing symmetric division (Fig. 1d, Additional file 2: Movie S1). The monitored AsPC1 cells had 70% symmetric, 25% asymmetric and 5% ambiguous (Data not shown). The monitored PANC1 cells had 80% symmetric, 10% asymmetric and 10% ambiguous (Data not shown). These observations suggest that both symmetric and asymmetric cell division transpire in PDA with symmetric division being more widespread.

RETRACTED

**Fig. 1:** PDA cells mostly divide symmetrically. **a** Schematic illustration of symmetric cell division (SCD) and asymmetric cell division (ACD) in low and high-grade tumorigenesis. **b** Frozen, human PDA tissue sections were stained for Notch (*green*), Numb (*red*) and counterstained with Dapi (*blue*). The Notch and Numb images were merged using FIJI software. The white arrows mark positive Notch staining on the proliferative sites. **c** Schematic illustration of SCD and ACD by time-lapse microscopy. **d** Established PDA cell lines were monitored by time-lapse microscopy under physiologic conditions for a period of 3 divisions and a total of 80 h. The number of visible cells is indicated on each slide



**Additional file 2: Movie S1.** A single AsPC1 cell was monitored over three replication cycles under physiologic conditions for about 80 h using time-lapse microscopy. The cells were re-focused periodically to avoid out-of-focus images. The images were processed using FIJI software. (MP4 1559 kb)


### Quercetin upregulates miR-200b-3p

To study a putative effect of quercetin, known to target pancreatic CSCs [35, 36], miR signaling and the mode of CSCs divisions, we performed a miR expression profiling of synchronized AsPC1 cells before and after treatment with quercetin for 12 h. The microarray data with the accession number E-MTAB-4718, was uploaded to Array Express and 105 miRs were found to be differentially expressed. Of these, 80 miRs were upregulated and 25 miRs were down-regulated (Fig. 2a). On the grounds that Notch signaling is implicated in CSCs’ fate determination, we performed *in silico* analyses, with interest to only the miRs out of the 105 differentially regulated that are involved in Notch signaling. This resulted to only 11 miRs namely; let-7c, miR-200a-3p, miR-200b-3p, miR-103a-3p, miR-1202, miR-125b-5p, miR-1268a, miR-6088, miR-3665, miR-4651 and miR-96-5p (Fig. 2a). The microarray data was validated by qRT-PCR analysis using six out of the 11 miRs (Fig. 2b).

**Fig. 2:** MiR-200b-3p could be a cell fate determinant miRNA. **a** *In silico* analyses was used to identify 11 out of 105 differentially regulated miRs, as players in Notch signaling/cell fate determination. **b** Using qRT-PCR, the microarray data was validated by Taqman® miRNA assay. RNA isolation from untreated (CO) and treated (Q, 50 μM) AsPC1 cells, followed by reverse transcription and PCR. RNU44 was used to normalize the expression levels and the average fold change of the CO was set to 1, while the expression level in the quercetin-treated cells was related to the control. **c** Human homolog of the segregating determinants. **d** Putative binding sites of miR-200b-3p in the 3’UTR of the segregating determinants (Numb, Prox1, and Trim2) and Notch1 was identified using TargetScan database. The seed-binding regions are marked in red. All assays were performed in triplicates, repeated at least three times and the means ± S.D. are shown. *P < 0.05, **P < 0.01

RETRACTED

### MiR-200b-3p as a cell fate determinant

To select the most important candidate miR from the 11, we performed a further in silico studies using the TargetScan® database to evaluate which of these miRs was predicted to target Notch and the human segregating determinants; Numb, Prox1 and Trim (Fig. 2c). MiR-200b-3p was identified as the only candidate (Fig. 2d, Additional file 3: Data 1), thus suggesting that this miR could be a cell fate determinant in PDA.

### MiR-200b-3p directly targets the Notch1 3’UTR

Considering that the segregating determinants, Numb, Prox1 and Trim directly or indirectly inhibits Notch, we opted to validate Notch1 as a direct target of miR-200b-3p. Whence, we performed a dual luciferase reporter assay using a commercially available renilla luciferase reporter construct expressing the Notch1 3’UTR. AsPC-1, AsanPaCa and PANC-1 cells were co-transfected with a reporter construct of the Notch1 3’ UTR or with control firefly plasmid together with either miR-200b-3p mimic or a miR non-coding control (miR-NC). Forty-eight hours after transfection, the luciferase activity was quantified in a luminescence microplate reader. We found a significantly reduced luciferase activity of the Notch1 reporter in the presence of miR-200b-3p, whereas no reduction of luciferase activity occurred with the empty vector control or in the presence of miR-NC (Fig. 3a). These results fitly show that Notch1 is a direct target gene for miR-200b-3p.

**Fig. 3:** MiR-200b-3p switches SCD to ACD. **a** MiR-200b-3p targeting the Notch1 mRNA through a targeting sequence located at the 3’UTR. Dual luciferase assay were performed to test the interaction of miR-200b-3p and its targeting sequence in the Notch1 3’UTR using constructs containing the predicted targeting sequence cloned into the 3’UTR of the reporter gene. Data represent three independent experiments with triplicate measurements. **b** AsPC1, AsanPaCa and PANC1 cells were transfected with 50 nM miR-200b-3p or miR-NC mimics or were treated with 50 μM quercetin (Q) or not (CO). Forty-eight-hours after transfection, the cells were utilized for Taqman® gene expression assays, quantifying Notch1 and Numb expressions. GAPDH served as control for equal conditions. **c** AsPC1 cells were treated as described above and total proteins obtained and analyzed by western blot. β-Actin served as controls for equal conditions. **d** AsPC1 cells transfected with 50 nM miR-200b-3p or miR-NC mimics were monitored by time-lapse microscopy under physiologic conditions for a period of 3 divisions. All assays were performed in triplicates, repeated at least three times and the mean ± S.D. are shown. *P < 0.05, **P < 0.01

RETRACTED

### MiR-200b-3p switches symmetric to asymmetric division

To establish the correlation between the observed down-regulation of miR-200b-3p and upregulation of Notch1 in control PDA cells, we quantified the mRNA and protein expressions of Notch1 and Numb. Our results show upregulation of Notch1 and down-regulation of Numb in control groups but a complete reversal of this phenomenon in miR-200b-3p and quercetin treated groups (Fig. 3b, c), indicating a possible switch from symmetric to asymmetric division. To validate this assumption, we performed a time-lapse microscopy, monitoring synchronized miR-NC and miR-200b-3p transfected AsPC1 cells for 3 division phases over 80 h. We observed that 75% of the control cells divided symmetrically, 20% asymmetrically and 5% ambiguously, while 60% of the miR-200b-3p-transfected cells divided asymmetrically, 30% symmetrically and 10% ambiguously (Fig. 3d). In toto, these results imply that miR-200b-3p switches the mode of CSCs division from symmetric to asymmetric.

### MiR-200b-3p inhibits CSCs self-renewal and proliferation

Next, we questioned if the switch from symmetric to asymmetric division is associated with CSCs self-renewal and proliferation. Hypothetically, symmetric division would result to more self-renewal and proliferation than ACD by inhibiting Notch signaling (Fig. 4a). Then, we performed serial tumorsphere propagation assays to evaluate the impact of miR-200b-3p on self-renewal and proliferation. Resuspended cells in tumorsphere medium were mixed in a ratio of 1:1 with matrigel and plated in a 24-well plate to avoid false positives and ensure that tumorspheres resulted from single CSCs and not from the aggregation of cells. Upon polymerization, the mixture was covered with unadorned tumorsphere medium (CO) or transfection mixture of the tumorsphere medium with 50nM of miR-NC/miR-200b-3p or 50 μM of quercetin in the tumorsphere medium. Subsequently, the resultant tumorspheres were passaged for three generations. MiR-200b-3p and quercetin significantly decreased tumorsphere formation (Fig. 4b). After being passaged for three generations, the ability to form new tumorspheres was practically lost in cells from the miR-200b-3p and quercetin treated groups whereas cells from the control groups (CO and miR-NC) significantly continued to form tumorspheres (Figs. 4b and 5a). These observations are in coherence with the switch from symmetric to asymmetric division by miR-200b-3p. Next, we evaluated the influence on proliferation by dissociating the tumorspheres from each group to single cells using trypsin-EDTA. The viable cells were then counted using the automated Z™ Series COULTER COUNTER® Cell and Particle Counter. Likewise, miR-200b-3p and quercetin tumorspheres had significantly lower cell numbers than the tumorspheres from the control groups (Fig. 5b). This therefore indicates that miR-200b-3p inhibits proliferation and it is consistent with the inhibition of self-renewal and hints of likely differentiation.

RETRACTED

**Fig. 4:** MiR-200b-3p inhibits CSCs self-renewal in vitro. **a** Schematic illustration of SCD and ACD with respect to self-renewal. Notch signaling and self-renewal are active in the both daughter cells in SCD. In ACD, notch signaling is activated in one and the other is inactive. **b** AsPC1, AsanPaCa and PANC1 cells in 1:1 mixture of tumorsphere medium and matrigel were seeded in a 24-well plate and allowed to polymerize. One milliliter of plain tumorsphere medium without treatment or 50 nM miR-NC transfection mixture or 50 nM miR-200b-2p transfection mixture or 50 μM quercetin was added to the CO, miR-NC, miR-200b-3p and Q groups respectively. The resulting tumorspheres were passaged for 3 generations

**Fig. 5:** MiR-200b-3p inhibits cell proliferation. **a** The number of tumorspheres from each generation was counted under a light microscope. **b** Trypsin-EDTA was used to dissociate the tumorspheres to single cells. The viable cells were counted using the automated Z™ Series COULTER COUNTER® Cell and Particle Counter. All assays were performed in triplicates, repeated at least three times and the mean ± S.D. are shown. *P < 0.05, **P < 0.01

### MiR-200b-3p triggers cell differentiation by inhibiting notch signaling

To substantiate the likelihood of differentiation, we cultured the dissociated tumorsphere cells in regular medium (DMEM, 10% FCS, 1% HEPES). The cells were left untransfected or treated with 50 μM quercetin or 50nM *mir*Vana™ mimics of miR-200b-3p or a miR-NC for every 72 h for a period of 12 days and subsequently evaluated for osteogenic, adipogenic and chrongenic differentiations. High heterogeneous expressions of osteoblasts, adipocytes and chondrocytes were detected in the miR-200b-3p and quercetin treated groups while little or no differentiation activity was detected in the control groups (Fig. 6a, b and c). These observations suggest that the differentiation is as a result of the inhibition of self-renewal (Additional file 4: Figure S2).

RETRACTED

**Fig. 6:** MiR-200b-3p triggers cell differentiation. **a** Dissociated AsPC1, AsanPaca and PANC1 cells were cultured in regular medium (DMEM, 10% FCS, 1% HEPES). The cells were treated with 50 nM of miR-200b-3p or miR control (miR-NC) mimics for 72 h or were treated with quercetin 50 μM for 12 h (Q) or were left untreated (CO) for every 72 h for a period of 12 days and subsequently evaluated for osteogenic differentiation. Heterogeneous osteogenic differentiation was detected using Sigma Fast BCIP/NBT substrate. The positive cells appear deep *bluish purple*. **b** Dissociated AsPC1, AsanPaca and PANC1 cells were treated as described above and evaluated for adipogenic differentiation. Heterogeneous adipocytes were *stained red* by the *Oil Red* O staining solution and visualized with a 10 × magnification using an inverted microscope **c** Dissociated AsPC1, AsanPaca and PANC1 cells were treated as described above and evaluated for chrondrogenic differentiation. Heterogeneous chondrogenic differentiation was detected as intense *dark-blue* coloration while the other cells were mostly *light bluish*. The bar indicates 100 μm

## Discussion

In this study, we show that highly aggressive PDA cells with CSC features can perform self-renewal by symmetric division; yielding two CSCs. In addition, the cells can divide asymmetrically; yielding a CSC and a differentiated non-CSC. However, the symmetric division mode was more prevalent. MiR-200b-3p plays a major role in the decision of a PDA cell to perform either symmetric or asymmetric division by modulating Notch signaling. And it putatively targets the segregating determinants. Hence, miR-200b-3p is suggested as a cell determinant miR in PDA.

Quercetin has been shown to inhibit pancreatic cancer growth and self-renewal [36, 37]. In our previous study, we demonstrated that miRs are robust alternatives to facilitate the delivery of quercetin mediated effects to patients, which otherwise is very challenging to be achieved by diet alone [24]. The miR-200 family of microRNAs made up of five members (miR-200a, miR-200b, miR-200c, miR-141 and miR-429) is an enforcer of the epithelial phenotype [38]. They are crucial players in cancer initiation, proliferation, migration, invasion and tumor growth [39]. MiR-200b in particular has been found to be involved in tumorigenesis and inhibition of tumor growth and cell fate control [40, 41].

Herein, we have shown that the expression of miR-200b is modulated by quercetin. Its expression is low in PDA cells and induced to higher levels upon quercetin treatment. This is the first time these findings have ever been identified. However, they are not surprising, owing to the fact that miR-200b is expressed at high levels in normal epithelial cells like the pancreas [42]. Thus, quercetin induces miR-200b expression in PDA cells in a bid to return it back to normalcy.

RETRACTED

Symmetric division was observed to be more prevalent in PDA cells and patient derived tissues. Remarkably, in the patient derived tissues, the symmetrically dividing cells were mainly observed in the pancreatic duct glands. The pancreatic ducts are known to possess stem cell niches and are the principal site of proliferation [43]. Symmetric division inevitably causes exponential cell division leading to tumor growth and progression.

An important factor in tumor growth and cell fate determination is the Notch signaling. Symmetric division gives rise to two identical cells in which the Notch signaling pathway is active in both of them. On the other hand, asymmetric gives rise to one cell in which the Notch signaling pathway becomes activated and one in which this pathway remains inactive. Notch acts by its ligand binding to its receptors causing the cleavage of Notch receptors and the resulting nuclear translocation of Notch intracellular domain (NICD) [44]. The difference in Notch signaling activity is established by Numb. Its functional role on cell fate decisions is exercised by antagonizing Notch signaling activities. This it does by the ubiquitination of the membrane bound Notch1 receptor consequently degrading its NICD upon receptor activation [17]. Our results show that the significantly higher expression of Notch compared to Numb, which occurred in PDA cells, is reversed by miR-200b-3p or quercetin. This observation, which suggests a switch from symmetric to asymmetric division, was further strengthened by our time-lapse microscopy analysis.

Apart from Numb, there are other proteins that are involved in cell fate determination like Prox1 and Trim. Together with Numb, they are known as human segregating determinants because their segregation into one of the two daughter cells results to distinct cell fates [45]. Our in silico analyses have shown that miR-200b putatively targets the segregating determinants. In line with our observations are studies that identified Trim as a regulator of asymmetric division, cellular differentiation and Notch signaling in CSCs [34]. Herein, they were critical in the decision to select miR-200b-3p as the most important miR candidate out the 11 miRs involved in Notch signaling.

To further understand the mechanism of the quercetin-induced miR-200b-3p regulation of the mode of self-renewal divisions, tumorspheres propagation assay was performed. Noteworthy inhibition of self-renewal by miR-200b-3p or quercetin was observed with concomitant decrease in proliferation. Further analyses of the resulting cells from the tumorspheres indicated immense differentiation of the cells by miR-200b-3p or quercetin. These results correspond to observations that elevated Numb levels support differentiation [46].

RETRACTED

## Conclusion

Taken together, we conclude that miR-200b-3p is down-regulated in PDA and its induction by quercetin may render the CSCs less aggressive by a switch of the cell division mode. MiR-200b-3p influences cell fate decisions in PDA by modulating Notch signaling. By reversing the elevated Notch levels with simultaneous decrease in Numb levels, inhibition of self-renewal and decrease of proliferation, it switches symmetric to asymmetric division. Hence, we propose miR-200b-3p as a cell fate determinant in PDA. Restoration of miR-200b-3p functions in cancer cells may represent an important therapeutic strategy for future cancer treatment.

## Additional files

Additional file 1: Figure S1. Double immunofluorescence staining was performed on 6-μm frozen pancreatic ductal adenocarcinoma patient tissue sections using mouse monoclonal anti-Cytokeratin, pan (Mixture) antibody (Sigma-Aldrich, USA), rabbit monoclonal anti-Notch1 antibody (Cell Signaling, Danvers, MA), goat polyclonal Numb antibody (Abcam, Cambridge, UK) and rabbit polyclonal Ki67 antibody (Abcam, Cambridge, UK). (PDF 15592 kb)
Additional file 3: Data 1 The binding sites of miR-200b-3p in the 3’UTR of Numb, Prox1, Trim2 and Notch1 were identified using TargetScan database. (XLSX 247 kb)
Additional file 4: Conditioned experiement was performed to confirm whether the effects of quercetin are due to the upregulation of miR-200b-3p, using eight conditions as follows: (1) Control, untreated cells (CO), (2) MiRNA negative control (miR-NC), (3) MiR-200b-3p inhibitor (miR-200b-), (4) MiR-200b-3p mimic (miR-200b+), (5) Quercetin (Q), (6) Quercetin plus miRNA negative control (Q+miR-NC), (7) Quercetin plus miR-200b-3p inhibitor (Q+miR-200b-), (8) Quercetin plus miR-200b-3p mimic (Q+miR-200b+). Pancreatic cancer cell line AsPC1 in the aforementioned treatment groups were evaluated for tumorsphere formation. The resulting tumorspheres were evaluated and thereafter dissociated into single cells and the cell numbers evaluated. The resulting cells were plated with DMEM + FCS + HEPES. After 72h of treatment as listed above, the cells were evaluated for osteogenic and chondrogenic differentiation. (PDF 188 kb)
